The article "A new approach to constructing confidence intervals for population means based on small samples" was retracted in 2023. Reason: compromised peer review.

# A new approach to constructing confidence intervals for population means based on small samples

**DOI:** 10.1371/journal.pone.0271163

**Published:** 2022-08-17

**Authors:** Hao-Chun Lu, Yan Xu, Tom Lu, Chun-Jung Huang

**Affiliations:** 1 Department of Management Science, National Yang Ming Chiao Tung University, Hsinchu, Taiwan; 2 Graduate Institute of Management, Chang Gung University, Taoyuan, Taiwan; 3 School of Mathematics, Ocean University of China, Qingdao, China; 4 Department of Mathematics and Statistics, Texas Tech University, Lubbock, Texas, United States of America; 5 Fab12 Manufacturing-1 Department, Taiwan Semiconductor Manufacturing Company, Hsinchu, Taiwan; University of New Mexico - Albuquerque: The University of New Mexico, UNITED STATES

## Abstract

This paper presents a new approach to constructing the confidence interval for the mean value of a population when the distribution is *unknown* and the sample size is *small*, called the Percentile Data Construction Method (PDCM). A simulation was conducted to compare the performance of the PDCM confidence interval with those generated by the Percentile Bootstrap (PB) and Normal Theory (NT) methods. Both the convergence probability and average interval width criterion are considered when seeking to find the best interval. The results show that the PDCM outperforms both the PB and NT methods when the sample size is less than 30 or a large population variance exists.

## 1. Introduction

Constructing the confidence interval (CI) for the mean value of an interesting population is a problem that can be found in numerous elementary statistics text books. When the distribution is unknown and the sample size is small (≤25 or 30), the usual approach is to use the *t* distribution to calculate the endpoints of an interval such that, while the interval is as narrow as possible it still contains the mean. This is termed the Normal Theory (NT) method for interval estimation. It can be formulated as follows:

$$\left(\bar{x}-t_{\left(1-\alpha )/2,(n-1\right)}(s/\sqrt{n}),\bar{x}+t_{\left(1-\alpha )/2,(n-1\right)}(s/\sqrt{n})\right)$$ (1)

where $\bar{x}$ is the sample mean, *s*^2^ is the sample variance, *n* is the sample size, and *α* is the confidence level. The NT interval relies on an assumption of normality. However, empirical evidence suggests that this may not be a valid assumption and could lead to erroneous conclusions. This makes it important to find an effective way of producing non-parametric estimates.

Bootstrap-based CI uses a re-sampling technique and is an effective alternative for estimating the mean because it works without any assumption of normality or other arbitrary patterns. In [1], a Percentile Bootstrap (PB) and a NT methods were used together to estimate audit values with small samples, which were randomly drawn from the gamma, log-normal, Weibull, and normal distributions. This approach produced better PB intervals than NT in terms of the convergence probability (CP) and average interval width (AIW) for a sample size of *n* between 30 and 200. In [2], the Standard Bootstrap (SB), Box–Cox transformation (BC), and NT methods were used to construct the CI for the mean of non-normal data with a sample size of *n* between 10 and 50. The conclusions of the study includes (1) the NT intervals had a better CP but a worse AIW than the SB and BC; (2) the SB appeared to generate a more valuable CI than the other two; (3) the sample size had an influence upon all three methods, especially SB. [3, 4] used five bootstrap-based estimators to construct the CI for the mean response time in *M*/*G*/1 and *G*/*G*/1 FCFS (First Come First Served) queuing systems, with sample sizes of *n* between 20 and 80. Here, the PB intervals were the best in terms of CP and AIW.

The article "A new approach to constructing confidence intervals for population means based on small samples" was retracted in 2023. Reason: compromised peer review.

Based on the above studies, it seems likely that the bootstrap technique is superior to other existing methods. However, when the sample size is very small it is doubtful whether the bootstrap technique will perform adequately. It has been shown that a sample size of at least 12 or 15 is necessary to ensure stable results using this approach [5]. As it is difficult, and even impossible in some cases to gain more reference data for analysis ([6–12]), the influence of very small samples remains a matter of concern.

[13, 14] developed a heuristic approach called the Data Construction Method (DCM) to create virtual data from limited patterns so that the size of available data could be enhanced. Numerical evidence showed that the DCM can improve the learning ability of a back propagation network (BPN) when an insufficient training data set is given. It has also proved to be capable of predicting the spatial distribution of severe earthquakes in Taiwan with reasonable accuracy [15]. In this paper, we apply DCM to calculate a percentile interval from generated virtual data to be able to estimate the mean when there are only small samples in hand. This approach, termed Percentile DCM (PDCM), can work without any assumptions regarding population distribution.

The rest of the paper is organized as follows: In Section 2, PDCM-related concepts and properties are introduced. Then, the PDCM algorithm is presented and explained by means of an illustrative example, followed by a sensitivity analysis. In Section 3, a simulation is used to compare the performance of PDCM, PB, and NT. A summary of the research, as well as the conclusions, is given in Section 4.

The article "A new approach to constructing confidence intervals for population means based on small samples" was retracted in 2023. Reason: compromised peer review.

## 2. Methodology

Before presenting the PDCM algorithm, we provide some information about its theoretical background in Section 2.1. In Section 2.2, the algorithm is presented after showing how the PDCM works. Then a numerical example is demonstrated in Section 2.3. A sensitivity analysis of PDCM’s parametric settings is then given in Section 2.4.

### 2.1 PDCM and its solution

Given a sample of data with size *n*, the sample can be described by a multiset as follows:

$$A_{o}=\left\{\left(a_{o_{i},},\lambda_{i}\right)|a_{o_{i}}\in \mathbb{R},a_{o_{i}}\leq a_{o_{i+1}},\lambda_{i}\in \mathbb{N},1\leq i\leq n,\sum_{i}\lambda_{i}=n\right\},$$ (2)

where $a_{o_{i}}$ is the element value, and *λ*_*i*_ is the corresponding frequency of $a_{o_{i}}$ in *A*_*o*_.

A representative mode of *A*_*o*_ is uniquely defined below:

**Definition 1** (*Sample mode*):

The mode of a sample can be taken to be:

$$\text{mode}\left(A_{o}\right)=\left\{\begin{array}{l} a_{o_{\left[n/2\right]}},\;\text{if}\;\lambda_{i}=1\;\text{for}\;\text{all}\;i;\\ \left\{\underset{a_{o_{i}}}{min}\left\{\underset{\lambda_{i}}{max}\left(a_{o_{i}},\lambda_{i}\right)\right\}\right\},\;o.w. \end{array}\right.$$ (3)

Based on Eq (3), *A*_*o*_ can be translated into:

$$A=\left\{\left(a_{i},\lambda_{i}\right)|a_{i}\in \mathbb{R},a_{i}\leq a_{i+1},\lambda_{i}\in \mathbb{N},1\leq i\leq n\right\},$$ (4)

where $a_{i}=a_{o_{i}}-\text{mode}(A_{o})$ and 0 ∈ *A*.

Now let us consider another multiset: *C* = {(1,1), (*c*,1)} where *c*>1. The multiset division of *A* by *C*, which is used for virtual data generation, can then be defined as specified below.

**Definition 2** (*Multiset division*):

The multiset division [15] can be described as follows:

$$Z^{t}\equiv A(:)C^{t}=\{(z_{q^{t}},f_{q^{t}})|z_{q^{t}}\in [a_{1},a_{n}],f_{q^{t}}\in \mathbb{N},1\leq q\leq Q\},\forall t\in \mathbb{N},Q\leq 2^{t}n,$$ (5)

where *t* is a variable to indicate the number of divisions, and *Z*^*t*^ is the resultant multiset after doing a specific number of divisions.

To determine the termination times of *t*, Chebyshev’s Inequality can be adopted as the stop condition for the division procedure, as described below.

**Lemma 1** (*Chebyshev’s inequality*):

Given a random variable *x* with a mean of *μ* and a finite variance of *σ*^2^, for any value *k* >1, we have *P* (|*x*-*μ*| ≤ *kσ*) > = 1-(1/*k*^2^). ■

Chebyshev’s inequality [16] enables us to estimate the amount of data that needs to fall into [*μ*-*kσ*, *μ*+*kσ*], such that the lower bound of the probability of data occurring is ensured. If *μ* and *σ*^2^ are unknown [17], suggests adopting the sample mean $\bar{x}$ and variance *s*^2^, given a sample set of size *n*. Thus, Chebyshev’s inequality can be modified as follows:

$$P\left(\left|x-\bar{x}\right|\leq \frac{ks(n+1)}{n}\right)\geq 1-{\left[(n+1)\left(k^{2}+n-1\right)\right]}^{-1}\left(nk^{2}\right).$$ (6)

This provides a means of defining the stop rule for the division process as below.

The article "A new approach to constructing confidence intervals for population means based on small samples" was retracted in 2023. Reason: compromised peer review.

**Lemma 2** (*The stop rule for multiset division*):

Based on Eq (6), for any value *k*>1, the stop rule can be defined using the following:

$$\theta =P(|z_{q^{t}}-{\bar{x}}^{t}|\leq \frac{k(N+1)}{N}s^{t})\geq w=1-{\left[(N+1)\left(k^{2}+N-1\right)\right]}^{-1}\left(Nk^{2}\right),$$ (7)

where $N=\Sigma_{q}f_{q^{t}}=2^{t}n$, ${\bar{x}}^{t}=N^{-1}\Sigma_{q}z_{q^{t}}f_{q^{t}}$, and $s^{t}={\left({\left(N-1\right)}^{-1}\sum {\left(z_{q^{t}}-{\bar{x}}^{t}\right)}^{2}\right)}^{0.5}$.

Suppose the confidence level is (1-*α*). If *θ* ≥ *w* ≥ (1-*α*) at *t* = *T*, the multiset division procedure is terminated; otherwise, it is repeated. ■

Note that the values of *k* and *α* have a significant effect upon how many divisions should occur. If *α* is increased or *k* is decreased, more divisions are needed. If *α* is decreased or *k* is increased, fewer divisions are needed.

If Eq (7) is satisfied when *t* = *T*, we can let $z_{q^{T}}^{'}=z_{q^{T}}+\text{mode}(A_{o})$, giving:

$$Z^{T^{\prime }}=\left\{\left(z_{q^{T},}^{\prime }f_{q^{T}}\right)|z_{q^{T}}^{\prime }\in \left[a_{o_{1}},a_{o_{n}}\right],z_{q^{T}}^{\prime }\leq z_{{\left(q+1\right)}^{T}}^{\prime },f_{q^{T}}\in \mathbb{N},1\leq q\leq Q\right\}$$ (8)

where *Z*^*T*′^ is a so-called virtual dataset. As proved in [15], *Z*^*T*′^ has the following important properties.

**Property 1** (*Measurable size of the virtual data*):

Given *Z*^*T*′^ and *A*_*o*_, we have $\Sigma f_{q^{T}}=2^{T}n$. ■

When *t* = *T*, the amount of the obtained virtual data is 2^*T*^-fold the amount of the collected sample. This property describes the fact that the amount of available data can be enhanced through multiset divisions.

**Property 2** (*Mode conservation*):

Given *Z*^*T*′^ and *A*_*o*_, we have mode(*Z*^*T*′^) = mode(*A*_*o*_). ■

This property describes the fact that the modes of the obtained virtual data and the collected sample are the same as each other. As a result, the most important element value will always be retained, regardless of how many multiset divisions conducted.

**Property 3** (*Bounds conservation*):

Given *Z*^T′^ and *A*_*o*_, we have $inf(Z^{T^{'}})=a_{o_{1}}$ and $sup(Z^{T^{'}})=a_{o_{n}}$. ■

This describes the fact that the obtained virtual data will always be bound by the domain values of the collected sample. This property enables us to avoid any possible prediction bias resulting from a situation being unbounded [18].

The article "A new approach to constructing confidence intervals for population means based on small samples" was retracted in 2023. Reason: compromised peer review.

So, using the *α*/2 and (1-*α*/2) percentage points of *Z*^*T*′^, the confidence interval for the population mean can be denoted as follows:

$$\text{CI}=\left(Z_{\left(\alpha /2\right)}^{T^{\prime }},Z_{\left(1-\alpha /2\right)}^{T^{\prime }}\right).$$ (9)

By way of example, the PDCM interval for *α* = 0.05 would be $\left(Z_{\left(2.5\%\right)}^{T^{\prime }},Z_{\left(97.5\%\right)}^{T^{\prime }}\right)$.

The foregoing definitions and properties together yield the algorithm described in the following section.

### 2.2 The PDCM algorithm

**Step 0**: Set *t* = 1 and a constant *α*, where 0<*α*<1;
**Step 1**: Input a sample $A_{o}=\left\{\left(a_{o_{i},},\lambda_{i}\right)|a_{o_{i}}\in \mathbb{R},a_{o_{i}}\leq a_{o_{i+1}},\lambda_{i}\in \mathbb{N},1\leq i\leq n,\Sigma_{i}\lambda_{i}=n\right\}$ and determine an arbitrary multiset *C* = {(1, 1), (*c*, 1)}, where *c*>1;
**Step 2**: If ∀*i*, *λ*_*i*_ = 1, $\text{mode}\left(A_{o}\right)=a_{o_{\left[n/2\right]}}$; otherwise, $\text{mode}\left(A_{o}\right)=\left\{\underset{a_{o}{}_{i}}{\text{min}}\left\{\underset{\lambda_{i}}{\text{max}}\left(a_{o}{}_{i},\lambda_{i}\right)\right\}\right\}$.
  Let $a_{i}=a_{o_{i}}-\text{mode}(A_{o})$. Then $A=\left\{\left(a_{i},\lambda_{i}\right)|a_{i}\in \mathbb{R},a_{i}\leq a_{i+1},\lambda_{i}\in \mathbb{N},1\leq i\leq n\right\}$.
**Step 3**: Let $Z^{t}\equiv A(:)C^{t}=\left\{\left(z_{q^{t}},f_{q^{t}}\right)|z_{q^{t}}\in [a_{1},\;a_{n}],f_{q^{t}}\in \mathbb{N},1\leq q\leq Q\right\}$.
**Step 4**: Set a constant *k*, where *k*>1, and confirm $\theta =P\left(\left|z_{q^{t}}-{\bar{x}}^{t}\right|\leq \frac{k(N+1)}{N}s^{t}\right)\geq w=1-{\left[(N+1)\left(k^{2}+N-1\right)\right]}^{-1}\left(Nk^{2}\right)$, where $N=\Sigma_{q}f_{q^{t}}=2^{t}n$, ${\bar{x}}^{t}=N^{-1}\Sigma_{q}z_{q^{t}}f_{q^{t}}$, and $s^{t}={\left({\left(N-1\right)}^{-1}\sum {\left(z_{q^{t}}-{\bar{x}}^{t}\right)}^{2}\right)}^{0.5}$.
  If *θ* ≥ *w* ≥ (1 − *α*) at *t* = *T*, go to Step 5; otherwise, set *t* = *t*+1 and go to Step 3;
**Step 5**: Assuming *t* = *T*, calculate $z_{q^{T}}^{'}=z_{q^{T}}+\text{mode}(A_{o})$ to output *Z*^*T*′^.
**Step 6**: Given the confidence level is (1-*α*), the confidence interval is $\left(Z_{\left(\alpha /2\right)}^{T^{\prime }},Z_{\left(1-\alpha /2\right)}^{T^{\prime }}\right)$.

In the next section we will provide an example to explain this algorithm in detail.

### 2.3 An illustrative example

This example refers to a notional accounting population and their accounts receivable. A random sample from an accounting firm in Taiwan is generated including the data for eight accounts receivable [2]: 510, 2684, 2907, 3165, 3553, 3640, 7267, 13571 (1 unit = 1,000 New Taiwan dollars). The PDCM algorithm using the data will proceed as follows:

**Step 0**: Set *t* = 1 and *α* = 0.05.
**Step 1**: Let this sample be denoted by *A*_*o*_ = {(510, 1), (2684, 1), (2907, 1), (3165, 1), (3553, 1), (3640, 1), (7267, 1), (13571, 1)}. Then, set *C* = {(1, 1), (1, 10)}.
**Step 2**: From Eq (3), mode(*A*_*o*_) = 3165 is used to transform *A*_*o*_ into *A* = {(-2655, 1), (-481, 1), (-258, 1), (0, 1), (388, 1), (475, 1), (4102, 1), (10406, 1)}.
**Step 3**: Let $Z^{t}\equiv A(:)C^{t}=\left\{\left(z_{q^{t}},f_{q^{t}}\right)\right\}$. Beginning at *t* = 1, we have
$$\begin{array}{ll} Z^{1} & \equiv A\left(:\right)C\;=\{\left(-2655,1\right),\;\left(-481,1\right),\;\left(-265.5,1\right),\;\left(-258,1\right),\;\left(-48.1,1\right),\;\left(-25.8,1\right),\;\left(0,2\right),\\ & \left(38.8,1\right),\;\left(47.5,1\right),\;\left(388,1\right),\;\left(410.2,1\right),\;\left(475,1\right),\;\left(1040.6,1\right),\;\left(4102,1\right),\;\left(10406,1\right)\}. \end{array}$$
  Similarly,
$$\begin{array}{ll} Z^{2} & \equiv A(:)C^{2}=[A(:)C](:)C=Z^{1}(:)C\\ & =\left\{\left(-2655,1\right),\left(-481,1\right),\left(-265.5,2\right),\left(-258,1\right),\left(-48.1,2\right),\left(-26.55,1\right),\left(-25.8,2\right),\left(-4.81,1\right),\right.\\ & \;\left(-2.58,1\right),\left(0,4\right),\left(3.88,1\right),\left(4.75,1\right),\left(38.8,2\right),\left(41.02,1\right),\left(47.5,2\right),\left(104.06,1\right),\left(388,1\right),\\ & \;\left.\left(410.2,2\right),\left(475,1\right),\left(1040.6,2\right),\left(4102,1\right),\left(10406,1\right)\right\}. \end{array}$$
**Step 4**: Set *k* = 2. As shown in Table 1, the division stop condition is satisfied at *t* = 4. Then we have the components of *Z*^4^ as follows:
$$\begin{array}{ll} Z^{4} & =\{(-2655,1),(-481,1),(-265.5,4),(-258,1),(-48.1,4),(-26.55,6),\cdots ,(0,16),\\ & \cdots ,(388,1),(410.2,4),(475,1),(1040.6,4),(4102,1),(10406,1)\}. \end{array}$$
  **Step 5**: Let $z_{q^{4}}^{'}=z_{q^{4}}+3165$. This provides for the generation of 128 virtual data points, as follows:
$$\begin{array}{ll} Z^{4^{\prime }} & =\{(510,1),(2684,1),(2899.5,4),(2907,1),(3116.9,4),(3138.45,6),\cdots ,(3165,16)\\ & \cdots ,(3553,1),(3575.2,4),(3640,1),(4205.6,4),(7267,1),(13571,1)\}. \end{array}$$
**Step 6**: Taking the 2.5% and 97.5% percentage points of *Z*^4′^ as the lower and upper interval limits, an interval of (2899.5, 4205.6) with a width of 1306.1 is obtained, on the basis of which the mean of the accounts receivable can be estimated.

**Table 1:** The results of the stopping condition of the division procedure.

*T*	${\bar{x}}^{t}$	*s* ^*t*^	*θ*	*w*	*θ* ≥ *w* ≥ 1 − *α* = 0.95
1	823.42	2776.18	0.94	0.80	No
2	452.88	2007.34	0.97	0.89	No
3	249.08	1440.97	0.95	0.94	No
4	136.996	1030.12	0.98	0.97	Yes

The above example demonstrates the simplicity of this approach to calculating the CI for the mean of an interesting population. As previously mentioned, PDCM works without any assumptions regarding the population distribution. Note also that the percentile intervals derived using PDCM are related to the values of *c* (at Step 1) and *k* (at Step 4). To elaborate upon how the correct setting of these two parameters was arrived at, the following section provides a sensitivity analysis.

The article "A new approach to constructing confidence intervals for population means based on small samples" was retracted in 2023. Reason: compromised peer review.

### 2.4 Sensitivity analysis for the values of *c* and *k*

Before undertaking the sensitivity analysis, the following two estimation performance indices that are generally used to assess CI quality were established.

**Definition 3** (*Convergence probability* (*CP*) & *average interval width* (*AIW*)):

Let *X*_1_, …, *X*_*n*_ denote a random sample from an unknown distribution and suppose that the interval $\left({\hat{\mu }}_{L},{\hat{\mu }}_{U}\right)$ is used to estimate the mean (*μ*). Let the data associated with the given sample of size *n* be drawn from the given population *P* times. The CP and AIW can then be defined as follows:

$$\text{CP}=Pr\left({\hat{\mu }}_{L,p}\leq \mu \leq {\hat{\mu }}_{U,p}|1\leq p\leq P\right),$$ (10)

$$\text{AIW}=\left[\Sigma_{p=1}^{p}({\hat{\mu }}_{U,p}-{\hat{\mu }}_{L,p})\right]/P.$$ (11)

where CP ∈ [0, 1] and $\text{AIW}\in {\mathbb{R}}^{+}$.

Using PDCM, Eqs (10) and (11) can be rewritten as follows:

$${\text{CP}}_{\text{PDCM}}=Pr\left(Z_{(\alpha /2),p}^{T^{\prime }}\leq \mu \leq Z_{(1-\alpha /2),p}^{T^{\prime }}|1\leq p\leq P\right),$$ (12)

$${\text{AIW}}_{\text{PDCM}}=\left[\Sigma_{p=1}^{p}(Z_{(1-\alpha /2),p}^{T^{\prime }}-Z_{(\alpha /2),p}^{T^{\prime }})\right]/P.$$ (13)

The larger the CP and the smaller the AIW, the better the quality of the CI, i.e. a higher CP delivers a more efficient CI and a narrower AIW delivers a more effective CI. These two indices were adopted because they are frequently used in practice to conduct evaluations for a variety of purposes. The AIW would be relatively important, for instance, when estimating the audit value of populations such as receipts, payments and assets [1]. For events such as nuclear power system accidents, severe earthquakes and tornados, the CP is often emphasized.

By observing various possible CP and AIW outcomes, a simulation was conducted to confirm whether the values of *c* and *k* really are correlated with the CI quality. Random samples from the following two distributions were considered:

$$\text{Normal}\left(\mu ,\sigma^{2}\right)={\left(\sqrt{2\pi }\sigma \right)}^{-1}exp\left[-\left(\frac{x-\mu }{2\sigma }\right)\right],x\in \mathbb{R},$$ (14)

$$\text{Gamma}(\gamma ,\beta )=\frac{{\left(x/\beta \right)}^{\alpha -1}exp(-x/\beta )}{\beta \Gamma (\gamma )},x\in {\mathbb{R}}^{+},$$ (15)

where the population mean and variance of Gamma(*γ*, *β*) are equal to *γβ* and *γβ*^2^, respectively. These two distributions play an important role in the modeling of quantitative phenomena in the natural and behavioral sciences and in industry. They also differ greatly in terms of skewness. For Eq (14), we defined *μ* = 1 and *σ*^2^ = 2, and for Eq (15) *γ* = 0.5 and *β* = 2, termed here as Normal(1,2) and Gamma(0.5,2). Thus, the population mean and variance for Normal(1,2) were the same as they were for Gamma(0.5,2), with the population mean, equaling 1, being what we wanted to estimate. For each distribution, there were 12 different sample sizes (*n*) to be considered, from 5 to 60, with a separation of 5. Over the course of the simulation, each number of random samples was processed 1000 times, indicated by *P* = 1000.

The article "A new approach to constructing confidence intervals for population means based on small samples" was retracted in 2023. Reason: compromised peer review.

The sensitivity analysis was conducted in relation to two cases: (1) letting *k* = 2 and *α* = 0.05 and then performing PDCM by setting *c* (from 10 to 300 with a separation of 10) and *n* (from 5 to 60 with a separation 5); (2) letting *c* = 10 and *α* = 0.05 and running PDCM by setting *k* (from 1.1 to 2.5 with a separation of 0.1) and *n* (from 5 to 60 with a separation of 5).

#### 2.4.1 Results of the sensitivity analysis for *c*

Figs 1 and 2, which cover four full contour plots, illustrate the variation in the mean estimation performance for Normal(1, 2) and Gamma(0.5, 2) in relation to the CP and AIW indices. If a contour plot is uniformly distributed at a specific sample size, this suggests that the performance is not correlated with the value of *c*.

**Fig 1:** The results of normal (1, 2) under *c* = 10~300, *n* = 5~60, *k* = 2, and *α* = 0.05.

**Fig 2:** The results of gamma (0.5, 2) under *c* = 10~300, *n* = 5~60, *k* = 2, and *α* = 0.05.

It can be seen from the four contour plots, there was no variation in the outcomes for CP and AIW at this specific sample size when different values of *c* were used to run the PDCM. Utilizing two-tailed Pearson tests, further statistical analysis showed that the value of *c* was not correlated with the outcomes for CP (p-value = 0.101) and AIW (p-value = 0.858) for the Normal(1,2) distributions. At the same time, the value of *c* was not correlated with the outcomes for CP (p-value = 0.973) and AIW (p-value = 0.864) for the Gamma(0.5,2) distributions. Thus, the value of *c* has an insignificant effect on the CI quality. This finding is supported by our previous research [15].

The article "A new approach to constructing confidence intervals for population means based on small samples" was retracted in 2023. Reason: compromised peer review.

#### 2.4.2 Results of the sensitivity analysis for *k*

The computational results are shown in Figs 3 and 4. In this case, if the contour plot is uniformly distributed at the specific sample size, this means that the CI quality for the CP and AIW outcomes is not correlated with the value of *k*.

**Fig 3:** The results of normal (1, 2) under *k* = 1.1~2.5, *n* = 5~60, *c* = 10, and *α* = 0.05.

**Fig 4:** The results of gamma (0.5, 2) under *k* = 1.1~2.5, *n* = 5~60, *c* = 10, and *α* = 0.05.

The four contour plots above show that changing the value of *k* has a significant effect on the outcomes for CP and AIW. Using two-tailed Pearson tests for further statistical analysis, it was found that *k* is significantly correlated with the outcomes for CP (p-value<0.001) and AIW (p-value<0.001) for the Normal(1,2) distributions. It is also significantly correlated with the outcomes of CP (p-value<0.001) and AIW (p-value<0.001) for the Gamma(0.5,2) distributions. Thus, the *k* value has a significant effect on the CI quality. Overall observations regarding how large the *k* value needs to be for the better CP and AIW outcomes are summarized in the following table:

Table 2 shows that the smaller the value of *k* the better the performance for AIW, while the bigger the value of *k* the better the performance for CP. Analysis of the PDCM intervals suggests that seeking a higher CP yet a smaller AIW is actually a trade-off.

**Table 2:** Suggested *k* value and the corresponding outcomes of CP and AIW.

Distributions	Referred plots	Suggested *k* value	Corresponding performance
Normal (1, 2)	Fig 3(a)	2.1≤*k*≤2.5	0.9≤CP≤1
	Fig 3(b)	1.1≤*k*≤1.7	0<AIW≤2
Gamma (0.5, 2)	Fig 4(a)	1.9≤*k*≤2.5	0.8≤CP≤1
	Fig 4(b)	1.1≤*k*≤1.4	0<AIW≤3

Figs 3 and 4 suggest that setting 1.1 ≤ *k* ≤ 2.5 for a simultaneously smaller AIW and a higher CP would be best when estimating the mean of Normal(1,2). If the CP index is preferred, we recommend *k* ≥ 2.1 for Normal(1,2) cases and *k* ≥ 1.9 for Gamma(0.5,2) cases.

Even if the population mean equaling 1 and variance equaling 2 are controlled, there is still a difference between the suggested *k* value for Normal(1,2) and Gamma(0.5,2). This may result from the fact that Normal(1,2) is a non-skewed model, while Gamma(0.5,2) is skewed. So, adjusting the *k* value for different populations is necessary when using the proposed algorithm. While the *k* value can be determined in advance, there is usually no prior information about the population distribution. Based on our experience, if the population distribution is unknown, we suggest using *k* = 2 to maintain a balance between the need for a larger CP and a smaller AIW.

The article "A new approach to constructing confidence intervals for population means based on small samples" was retracted in 2023. Reason: compromised peer review.

The results of the sensitivity analysis have confirmed that, while the *c* value has no impact, the *k* value has an important effect upon the CI quality. In the next section, we use the results of a comparative study to demonstrate the capacity of PDCM for estimating the population mean with small samples.

## 3. Comparative studies

The efficiency and effectiveness of PDCM at estimating population means with small samples were assessed by undertaking an experimental Monte Carlo simulation. As may be recalled from earlier, the benchmarks against which PDCM needs to be compared are the Normal Theory (NT) and Percentile Bootstrap (PB) methods. For the purposes of this comparison we again used CP and AIW. Before turning to the comparative study, let us briefly introduce NT and PB in greater detail:

- The Normal Theory method (NT)
  If we let *X*_1_, …, *X*_*n*_ be a random sample from an unknown distribution, then, if a dataset of size *n* is randomly drawn *P* times for each sample, the sample mean, ${\bar{x}}_{p}$, and standard deviation, *s*_*p*_, where 1≤*p*≤*P*, can be obtained. If the population mean (*μ*) falls exactly within the interval denoted by Eq (1), it is considered a success. Thus, the NT interval can be evaluated using the CP and AIW indices as follows:
$${\text{CP}}_{\text{NT}}=Pr\left({\bar{x}}_{p}-t_{\left(1-\alpha )/2,(n-1\right)}\left(s_{p}/\sqrt{n}\right)\leq \mu \leq {\bar{x}}_{p}+t_{\left(1-\alpha )/2,(n-1\right)}\left(s_{p}/\sqrt{n}\right)|1\leq p\leq P\right)$$ (16)
$${\text{AIW}}_{\text{NT}}=\left(2\Sigma_{p=1}^{p}t_{\left(1-\alpha )/2,(n-1\right)}\left(s_{p}/\sqrt{n}\right)\right)/P$$ (17)
- The Percentile Bootstrap method (PB)

The process used to apply PB to estimate a population mean is illustrated below:

1. Construct an empirical probability distribution, Ω, from a sample by placing a probability of 1/*n* at each point, *X*_1_, …, *X*_*n*_. This ensures that each sample element will have the same probability;
2. From Ω, draw a random sample of size *n* as a replacement, which is a “resample”;
3. Calculate the average of this resample, yielding μ*;
4. Repeat steps (2) and (3) *B* times, where *B* is a large number, to create a total of *B* resamples. The actual size of *B* will depend upon the tests to be run on the data. Typically, *B* = 1000 is required;
5. Given ${\hat{\mu }}_{1}^{*},{\hat{\mu }}_{2}^{*},\cdots ,{\hat{\mu }}_{B}^{*}$, the PB interval for *μ* can be calculated using the 100(1-*α*) percentile of the *B* resamples, as denoted by $\left({\hat{\mu }}_{\left(\alpha /2\right)}^{*},{\hat{\mu }}_{\left(1-\alpha /2\right)}^{*}\right)$.
6. Draw a random sample of size *n* from an unknown distribution *P* times and, here, the CP and AIW indices can be defined using the following:
$${\text{CP}}_{\text{PB}}=Pr\left({\hat{\mu }}_{(\alpha /2),p}^{*}\leq \mu \leq {\hat{\mu }}_{(1-\alpha /2),p}^{*}|1\leq p\leq P\right)$$ (18)
$${\text{AIW}}_{\text{PB}}=\left(\Sigma_{p=1}^{p}({\hat{\mu }}_{(1-\alpha /2),p}^{*}-{\hat{\mu }}_{(\alpha /2),p}^{*})\right)/P$$ (19)

The article "A new approach to constructing confidence intervals for population means based on small samples" was retracted in 2023. Reason: compromised peer review.

### 3.1 Description of the experiment

As in Section 2.4, this experiment focused on the Normal and Gamma distributions. For each distribution, we fixed the population mean at 1 and used 6 different population variances from 2 to 12 with a separation of 2. Meanwhile, random samples of 12 different sizes, from 5 to 60 with a separation of 5, were drawn from the specific population. The confidence level was 95%. So, we were interested in estimating the population mean, equal to 1, over a total of 144 cases (2 distributions × 6 populations per distribution × 12 sample sizes per population).

There were also some parametric settings to be prepared. Firstly, random samples for each specific sample size were generated 1000 times (*P*) using the functions *normrnd* and *gamrnd* provided by MATLAB 6.5. Secondly, *B* = 1000 was set for the PB. Thirdly, *c* = 10 was set for the PDCM because, as proved above, the *c* value is not correlated with the outcomes of CP and AIW. Fourthly, when using the PDCM we adopted *k* = 2 for the Normal cases and *k* = 1.5 for the Gamma cases. The overall simulation results, showing the CP and AIW outcomes, were then recorded for comparison.

### 3.2 Results of the experiment

The simulation results for the Normal distribution are presented in Table 3 and for the Gamma distribution in Table 4. To clearly demonstrate the comparison between NT, PB, and PDCM, the simulation results are summarized according to the following two circumstances.

**Circumstance 1**: the PDCM outperforms the PB or NT for interval estimation when using the CP index.
**Circumstance 2**: the PDCM outperforms the PB or NT for interval estimation when using the AIW index.

**Table 3:** The results of normal cases under the CP and AIW indices.

			*n* = 5	*n* = 10	*n* = 15	*n* = 20	*n* = 25	*n* = 30	*n* = 35	*n* = 40	*n* = 45	*n* = 50	*n* = 55	*n* = 60
**σ**^**2**^ **= 2**	**PB**	CP (%)	89.0	92.4	91.3	93.5	93.4	92.4	94.3	94.0	93.9	92.9	93.5	94.8
		AIW	1.73	1.34	1.14	1.00	0.90	0.82	0.76	0.72	0.68	0.64	0.61	0.59
	**NT**	CP (%)	88.7	90.1	87.1	89.8	90.1	89.0	90.7	89.7	89.9	88.6	89.3	91.9
		AIW	2.39	1.57	1.26	1.08	0.96	0.87	0.80	0.75	0.71	0.67	0.63	0.61
	**PDCM**	CP (%)	81.8	91.5	87.5	95.5	96.3	98.3	98.6	99.2	99.5	99.7	99.7	100.0
		AIW	2.73	1.61	0.79	0.33	0.36	0.39	0.47	0.45	0.32	0.33	0.45	0.38
**σ**^**2**^ **= 4**	**PB**	CP (%)	90.5	92.2	91.1	94.7	93.7	94.0	94.5	94.8	93.7	93.3	94.9	93.6
		AIW	2.50	1.88	1.61	1.42	1.26	1.16	1.08	1.01	0.96	0.91	0.87	0.83
	**NT**	CP (%)	90.0	88.9	88.5	91.1	89.7	90.8	89.2	91.0	91.2	90.5	90.9	90.9
		AIW	3.44	2.20	1.78	1.54	1.35	1.22	1.13	1.05	1.00	0.94	0.90	0.86
	**PDCM**	CP (%)	80.3	91.6	90.3	94.1	96.3	97.5	98.8	98.9	99.5	99.8	99.8	100.0
		AIW	3.31	1.60	0.39	0.51	0.48	0.63	0.58	0.53	0.55	0.45	0.53	0.50
**σ**^**2**^ **= 6**	**PB**	CP (%)	89.1	91.9	92.2	93.3	94.4	93.8	94.4	95.0	94.9	94.4	95.4	94.7
		AIW	3.04	2.33	1.99	1.73	1.55	1.44	1.34	1.25	1.18	1.12	1.07	1.03
	**NT**	CP (%)	88.8	91.1	89.7	89.4	89.2	90.7	90.5	91.4	90.3	90.3	90.9	89.6
		AIW	4.19	2.72	2.20	1.85	1.65	1.51	1.40	1.30	1.22	1.15	1.11	1.05
	**PDCM**	CP (%)	80.1	91.7	88.0	95.5	96.2	98.3	99.4	99.6	99.6	99.7	99.7	99.8
		AIW	1.99	1.20	0.90	0.63	0.78	0.62	0.69	0.63	0.62	0.52	0.61	0.62
**σ**^**2**^ **= 8**	**PB**	CP (%)	89.2	91.6	93.1	93.6	92.1	94.6	93.4	95.3	93.2	94.5	94.1	92.6
		AIW	3.42	2.70	2.29	1.98	1.82	1.63	1.53	1.44	1.37	1.29	1.23	1.18
	**NT**	CP (%)	86.9	88.8	90.7	88.8	88.5	92.0	88.6	91.6	89.4	90.2	90.4	88.8
		AIW	4.71	3.16	2.52	2.15	1.93	1.73	1.60	1.51	1.42	1.33	1.27	1.21
	**PDCM**	CP (%)	81.5	91.3	87.8	94.0	96.2	97.6	98.5	99.3	99.8	99.8	99.8	100.0
		AIW	0.82	0.48	0.56	0.64	0.73	0.94	0.91	0.87	0.97	0.99	0.71	0.80
**σ**^**2**^ **= 10**	**PB**	CP (%)	89.7	91.7	92.2	94.1	94.6	94.0	94.6	94.7	94.7	93.6	92.7	94.0
		AIW	3.84	3.02	2.52	2.24	2.03	1.84	1.71	1.62	1.52	1.45	1.38	1.32
	**NT**	CP (%)	89.7	89.4	88.3	90.4	91.0	90.1	91.1	90.2	91.5	90.0	89.7	89.6
		AIW	5.27	3.52	2.80	2.42	2.15	1.93	1.80	1.68	1.57	1.50	1.42	1.36
	**PDCM**	CP (%)	80.9	91.1	87.9	94.7	95.6	98.0	98.7	99.3	99.7	99.4	100.0	100.0
		AIW	1.19	0.92	0.68	0.82	0.82	0.98	1.03	1.13	0.88	0.83	0.88	0.77
**σ**^**2**^ **= 12**	**PB**	CP (%)	88.3	90.7	92.2	94.6	94.0	93.4	94.2	93.4	95.0	94.1	94.4	93.6
		AIW	4.32	3.24	2.80	2.43	2.21	2.03	1.87	1.77	1.66	1.58	1.51	1.44
	**NT**	CP (%)	89.2	88.8	90.2	90.5	89.2	89.6	90.3	89.0	92.1	88.3	90.6	90.1
		AIW	5.92	3.77	3.09	2.62	2.35	2.14	1.96	1.84	1.71	1.64	1.56	1.48
	**PDCM**	CP (%)	79.8	90.5	87.4	95.9	96.1	97.7	98.6	99.4	99.6	99.8	99.9	100.0
		AIW	0.86	0.53	0.94	1.08	0.98	1.07	1.03	1.08	1.10	0.92	1.23	0.83

The article "A new approach to constructing confidence intervals for population means based on small samples" was retracted in 2023. Reason: compromised peer review.

**Table 4:** The results of gamma cases under the CP and AIW indices.

			*n* = 5	*n* = 10	*n* = 15	*n* = 20	*n* = 25	*n* = 30	*n* = 35	*n* = 40	*n* = 45	*n* = 50	*n* = 55	*n* = 60
**σ**^**2**^ **= 2**	**PB**	CP (%)	57.7	68.2	70.2	75.0	74.0	78.5	76.7	81.3	80.1	81.2	81.8	80.8
		AIW	1.14	0.99	0.91	0.87	0.74	0.73	0.67	0.66	0.62	0.60	0.60	0.56
	**NT**	CP (%)	61.9	69.2	70.5	74.0	73.4	76.1	77.5	80.2	79.0	80.6	80.8	79.8
		AIW	1.63	1.20	1.03	0.96	0.80	0.79	0.72	0.70	0.65	0.63	0.63	0.59
	**PDCM**	CP (%)	69.9	88.3	88.2	93.2	91.2	94.0	95.0	96.9	95.7	97.4	97.1	98.1
		AIW	0.15	1.12	0.65	0.97	0.47	0.69	0.52	0.70	0.53	0.70	0.52	0.65
**σ**^**2**^ **= 4**	**PB**	CP (%)	54.6	64.4	66.4	68.8	74.7	75.9	76.5	75.7	77.9	80.5	79.5	79.2
		AIW	1.14	1.11	0.98	0.88	0.86	0.77	0.77	0.71	0.68	0.67	0.63	0.60
	**NT**	CP (%)	57.9	65.3	66.7	68.8	73.4	75.0	76.4	74.6	75.9	78.6	78.0	77.7
		AIW	1.65	1.33	1.13	0.98	0.94	0.83	0.83	0.76	0.72	0.70	0.67	0.62
	**PDCM**	CP (%)	69.3	89.1	93.2	96.7	97.0	98.2	99.1	99.3	99.4	99.7	99.9	99.9
		AIW	0.89	2.43	1.96	2.32	1.81	1.86	1.72	2.10	1.72	1.87	1.67	1.89
**σ**^**2**^ **= 6**	**PB**	CP (%)	52.5	60.0	64.7	69.5	71.7	74.2	74.2	73.9	77.3	77.1	76.8	79.5
		AIW	1.32	1.10	1.08	0.97	0.90	0.88	0.82	0.80	0.77	0.70	0.69	0.68
	**NT**	CP (%)	56.1	61.7	65.3	69.6	70.9	73.0	72.7	73.0	75.9	75.6	75.6	78.3
		AIW	1.90	1.34	1.24	1.08	0.98	0.96	0.87	0.86	0.82	0.73	0.72	0.72
	**PDCM**	CP (%)	67.3	88.0	93.0	96.4	98.0	98.1	98.4	99.5	99.8	99.4	99.6	100.0
		AIW	1.39	3.04	2.83	3.22	2.71	2.86	2.48	2.78	2.29	2.68	2.51	2.68
**σ**^**2**^ **= 8**	**PB**	CP (%)	48.3	57.0	68.0	67.9	70.1	71.6	74.2	72.1	75.9	77.8	78.1	77.4
		AIW	1.44	1.24	1.21	1.16	1.00	1.02	0.90	0.88	0.89	0.85	0.83	0.78
	**NT**	CP (%)	51.6	57.5	68.1	67.8	69.0	71.3	73.6	70.7	74.4	76.2	76.5	75.6
		AIW	2.07	1.52	1.39	1.29	1.09	1.10	0.96	0.93	0.94	0.90	0.87	0.82
	**PDCM**	CP (%)	61.4	85.9	91.6	95.1	97.0	96.8	98.4	99.4	99.3	99.4	99.8	99.9
		AIW	1.52	4.09	3.41	3.92	3.21	3.25	3.03	3.70	3.08	3.17	2.94	3.18
**σ**^**2**^ **= 10**	**PB**	CP (%)	49.6	58.5	62.5	67.6	67.3	72.3	71.5	72.7	74.3	76.2	75.5	76.9
		AIW	1.62	1.53	1.39	1.25	1.20	1.16	1.06	1.02	1.01	1.03	0.96	0.91
	**NT**	CP (%)	52.6	60.5	62.0	66.3	67.0	70.9	69.7	71.6	73.2	75.6	74.4	76.6
		AIW	2.34	1.87	1.60	1.40	1.33	1.27	1.14	1.09	1.07	1.08	1.01	0.95
	**PDCM**	CP (%)	58.2	84.2	88.3	93.5	96.5	96.7	98.5	98.4	98.3	99.6	99.2	100.0
		AIW	1.86	4.64	4.04	4.52	3.95	3.40	3.27	3.69	3.38	3.85	3.39	3.65
**σ**^**2**^ **= 12**	**PB**	CP (%)	44.5	58.2	61.1	64.6	65.3	68.2	69.2	71.9	73.3	72.7	73.2	74.5
		AIW	1.67	1.73	1.59	1.48	1.37	1.35	1.25	1.24	1.16	1.16	1.12	1.10
	**NT**	CP (%)	47.6	59.2	61.2	63.9	64.6	67.7	68.5	71.7	71.8	71.6	71.3	73.3
		AIW	2.47	2.13	1.84	1.66	1.51	1.48	1.35	1.34	1.25	1.23	1.18	1.16
	**PDCM**	CP (%)	58.3	81.6	88.1	92.4	95.2	96.6	97.0	98.6	98.7	99.0	99.3	99.6
		AIW	2.36	4.75	4.51	5.37	4.11	4.10	3.81	4.29	3.94	3.87	3.56	3.97

#### 3.2.1 Proportion of circumstance 1 with respect to different distributions, sample sizes and variances

For each of the circumstances, the comparative results will be discussed according to different population distributions, sample sizes, and population variances.

Fig 5 shows the proportion of Circumstance 1 with respect to the PDCM vs. the PB method and the PDCM vs. the NT method for each population distribution. The results show that, for the Normal distribution, the PDCM performed better than the PB and NT methods by up to 74% and 86%, respectively. For the Gamma distribution, the PDCM performed were better than the PB and NT methods by up 93% and 90%, respectively. As expected, the NT method performed better when estimating the Normal populations, where normality is assumed. In this study, the PDCM appeared to be superior to the NT method.

The article "A new approach to constructing confidence intervals for population means based on small samples" was retracted in 2023. Reason: compromised peer review.

**Fig 5:** Proportion of circumstance 1 for different distributions.

The comparative results for twelve different sample sizes are shown in Fig 6. The proportion of Circumstance 1 with respect to the PDCM vs. the PB method as well as the PDCM vs. the NT method was computed for each sample size. The results show that, outside of where *n* = 5 and *n* = 15, the PDCM completely outperformed the other two methods.

**Fig 6:** Proportion of circumstance 1 for different sample sizes.

In Fig 7, the comparative results for six different population variances are shown. The proportion of Circumstance 1 with respect to the PDCM vs. the PB method as well as the PDCM vs. the NT method was calculated for each population variance. In this case, PDCM outperformed the other two methods by an average ratio of around 80%. So, the PDCM generally offered a substantially better performance, especially as the variances increased.

**Fig 7:** Proportion of circumstance 1 for different variances.

#### 3.2.2 Proportion of circumstance 2 with respect to different distributions, sample sizes and variances

The proportion of Circumstance 2 discussed in this section relates to the performance of the three methods regarding the AIW index. When the results of Tables 3 and 4 are combined and compared for the PB and NT methods and the PDCM, the results can be summarized across the three dimensions of population distribution, sample size, and population variance. This provides for an analysis of the variations in estimation performance in relation to the AIW index.

In Fig 8, the performance of the PDCM was better than that of the PB or NT methods regarding the proportion of Circumstance 2 by 96% and 97%, respectively. For the Gamma population distribution, the performance of the PDCM was better than the PB and NT methods by 51% and 53%, respectively. The PDCM also appeared to be superior for the Normal distribution when considering both the CP and AIW indices.

**Fig 8:** Proportion of circumstance 2 for different distributions.

A further evaluation of Circumstance 2 across twelve different sample sizes is shown in Fig 9. Here, the PDCM performed noticeably better when the sample size was less than 30. When the sample size increased, the ratios of the AIW values decreased. So the advantage of using the PDCM also decreased.

The article "A new approach to constructing confidence intervals for population means based on small samples" was retracted in 2023. Reason: compromised peer review.

**Fig 9:** Proportion of circumstance 2 for different sample sizes.

Fig 10 shows the comparative results for six different population variances, with the proportion of Circumstance 2 being calculated with respect to the PDCM vs. the PB method and the PDCM vs. the NT method for each population variance. Here, the values for Circumstance 2 were more than 60% better for the PDCM, once again confirming its superiority to the PB and NT methods. The larger the variance, the better the AIW index for the PDCM.

**Fig 10:** Proportion of circumstance 2 for different variances.

Finally, when evaluating the proportions of both Circumstances 1 and 2 with respect to the Normal and Gamma distributions, the PDCM performance was superior to the PB method by 67% and 50%, respectively, and it was superior to the NT method by 72% and 56%, respectively. Taking an opposite perspective, in relation to the Normal and Gamma distributions, the PDCM performance was inferior to the PB method across all 72 trials by only 7% and 3%, respectively, and it was inferior to the NT method by just 1% and 1%, respectively.

## 4. Summary and discussion

To construct the confidence interval from small sample sets for the mean value of an interesting population, this paper has proposed the Percentile Data Construction Method (PDCM) that has its origins in the 1-DCM algorithm [15]. To validate the PDCM, a comparative study was conducted where its performance was compared to the Normal Theory (NT) and Percentile Bootstrap (PB) methods. The study was performed with simulations that were based on 144 instances across 2 distributions (Normal and Gamma), 6 population variances (*σ*^2^ = 2, 4, 6, 8, 10, and 12), 12 sample sizes (*n* = 5, 10, 15, 20, 25, 30, 35, 40, 45, 50, 55, and 60) and a confidence level of 1-*α* = 95%. The simulation results were evaluated using the average interval width (AIW) and convergence probability (CP) indices because these indices are often used in practice for different kinds of evaluation.

It was found that, depending on the CP, the PDCM was superior to the PB and NT methods for more than 80% of the 144 instances, and it performed especially well when the sample sizes were more than 20. The PDCM displayed a better performance than the PB and NT methods for at least 80% of the Normal distributions and approximately 60% of the Gamma distributions, in particular when the sample size was less than 30 or there was a larger population variance. Taking the CP and AIW indexes together, the PB method performed better than the PDCM in only one instance (with a sample size of 5 for the Normal(1,6) distribution), while the PB method itself outperformed the NT method across all the 144 instances considered. Based on computations carried out by a PC with an Intel^®^ Core^™^ i5 processor, 4GMB RAM, and a Windows 7 operating system, the PDCM and the PB method required approximately 40 and 1200 seconds, respectively, to perform their calculations. Thus, the PDCM was also found to be more efficient than the PB method in terms of computational cost. Our method does not need the parametric assumption. Therefore, even if the first moment of data generating distribution does not exist the proposed method still works well. Further simulation studies are still needed to consider other population distributions and variances and to compare the PDCM more broadly with bootstrap techniques.

The article "A new approach to constructing confidence intervals for population means based on small samples" was retracted in 2023. Reason: compromised peer review.

Regarding its applicability, a good estimator should possess high performance indices for both AIW and CP. However, different application contexts may allow for just one or the other of these two indexes to be adopted. For example, the AIW may be more important when estimating the audit value of populations such as receipts, payments and assets, while for events such as nuclear power system accidents, severe earthquakes and tornados, the CP is often emphasized. Our proposed procedure is flexible. As shown in Section 4.2.2, the *k* value can be adjusted to meet desired CP and AIW outcomes. When a larger *k* is set, a higher CP can be acquired. On other occasions, a larger AIW can be obtained for inference.

The authors wish to thank the Area Editor, the Associate Editor, and the anonymous referees for providing insightful comments and suggestions, which have helped us to improve the quality of the paper.
